RETRACTED

# Ligament Repair Method for Sports Dancers Based on Health Monitoring

**DOI:** 10.1155/2022/4369207

**Published:** 2022-09-14

**Authors:** Jijin Sun, Yan Sheng

**Affiliations:** ^1^College of Education, Qiongtai Normal University, Haikou 571127, Hainan, China; ^2^College of P. E, Qiongtai Normal University, Haikou 571127, Hainan, China

## Abstract

In sports dance training, the injury rate of athletes' ligaments is higher than that of ordinary ones. Careful study of ligament repair methods can better prolong the sports life of sports dance athletes. The purpose of this paper is to investigate how to analyze ligament repair in sports dancers based on health monitoring. This paper proposes a deep learning algorithm based on health monitoring and a neural network algorithm, both of which have the function of prediction. The experimental results of this paper show that the common injuries in sports dance include ankle ligament injury, medial and lateral knee ligament strain, lumbar muscle strain, toe joint strain, shoulder deltoid strain and other injuries. Among them, the number of ankle ligament injuries is the largest, with 36 people, accounting for 30%. The number of people with medial and lateral ligament strains in the knee joint ranks second with 32 people, accounting for 26%. The total proportion of two kinds of ligament strains is 56%, accounting for more than half. It can be seen that ligament strains are the most common in sports dance injuries, so it is of great research significance to repair the ligaments of sports dancers based on health monitoring.

## 1. Introduction

In the field of injury and rehabilitation of sports dancers, people have begun to pay attention to the repair of ligament injuries. For the normal growth and development of an athlete, ligament injury not only affects the training quality of the system, but also affects the normal level of the athlete's training and performance in competitions. This will lead to the decline of athletes' athletic ability, and even lead some elite athletes to end their sports career prematurely. After ligament injury, if the injury is very serious, the ligament is completely ruptured, and there is no active surgical treatment, the joint stability will be relatively poor in the later stage, which will lead to the occurrence of traumatic arthritis in patients.

Health monitoring is a survey that regularly observes the health status or irregularities of a specific population or sample of the population. Health monitoring in the process of health management refers to the regular and uninterrupted observation of these health risk factors in order to grasp the health and disease status of a specific target group or individual. Health monitoring can take the form of daily health monitoring, health services, and special services. Monitoring health status is a new approach to self-protection, moving from passive treatment to active examination, and potentially from passive treatment to active disease prevention. Because it can be detected early through regular monitoring, medical experts believe that even people who are healthy at first glance must be monitored every year or at least every 2 years.

RETRACTED

The innovations of this paper are: (1) This paper introduces the relevant theoretical knowledge of health monitoring and ligament repair of sports dancers, and proposes a deep learning algorithm based on health monitoring, and analyzes how the deep learning algorithm plays a role in the ligament repair of sports dancers. (2) This paper studies the ligament injury of 120 sports dancers. It can be known through experiments that health monitoring can be more beneficial to the ligament repair of sports dancers.

## 2. Related Work

As more and more attention has been paid to sports dance in recent years, the development of sports dance has also begun to develop rapidly. But in sports dance, it is easy to cause ligament damage. Heusdens et al. found that there is a great deal of interest in primary repair of the anterior cruciate ligament (ACL). Repair of ACL ruptures can be accomplished with separate suture tapes as well as reinforced ACL repair techniques. Their aim was to describe this ACL repair technique through video illustrations [1]. Guelfi et al. found that chronic ankle instability is defined as instability that persists for more than 6 months and requires surgery to stabilize the condition in the event of failure of comprehensive conservative treatment. They described arthroscopic lateral ligament repair and the use of these procedures is gaining popularity. Their main objective was to summarize and compare some methods of repairing ligaments [2]. Francisco et al. found that the size of the graft in cruciate ligament (ACL) surgery was strongly related to the chance of successful surgery. They also found that folding the graft smaller would make the operation smoother, and this simple method has been used by many doctors to achieve the purpose of their successful operation [3]. Tan et al. found that despite the introduction of minimally invasive methods, intraoperative bleeding remains a major risk in ligament reconstruction (ACLR) surgery. Through research, it has been analyzed that tranexamic acid (TXA) can effectively solve the problem of bleeding, which can minimize the complications of postoperative hemoarthrosis [4]. Shu et al. presented two cases of posterior cruciate ligament (PCL) repair using suture augmentation (SA) in the setting of multiligamentous knee injuries. Excellent clinical outcomes were achieved at two years of follow-up, with two patients returning to sports after injury. Both patients showed improvement in knee injury and the Osteoarthritis Outcome Score (KOOS) [5]. Tomoyuki et al aimed to determine the safe anchor insertion angle of the anterior talofibular ligament (ATFL) and calcaneofibular ligament (CFL) on CT images for minimally invasive repair of ATFL and CFL. To this end, they conducted related experiments [6].

RETRACTED

In the era of the prevalence of sports dance, sports dance athletes have become more diligent in training in order to improve their abilities, but this also leads to sports injuries that are prone to occur in sports dance training. If the injury is more serious, it will seriously affect the dancer's dance career, resulting in irreversible consequences. Therefore, it is necessary to use modern technology to monitor the health of the ligament repair of sports dancers, so as to help the athletes recover and return to the field as soon as possible. However, in traditional treatment, athletes generally have a wrong understanding of their own ligament repair. The above scholars have also proposed various methods of repairing ligaments, but they have not been able to adapt to the current era of big data intelligence. In order to make the ligament repair of sports dancers more correct and effective, intelligent health monitoring should be used.

## 3. Deep Learning Algorithm Based on Health Monitoring

### 3.1. Factors of Ligament Strain in Sports Dance

Sports dance, also known as international standard ballroom dance, is one of the sports events. It is a walking pas de deux competition accompanied by men and women. Sports dance has unique decorative and dance artistic value. Whether it is a dance arts program or a sports program, dance sports fully integrate recreation, fitness, performance, and competition. Its unique dance, passionate and changing music, and gorgeous costumes are loved and pursued by people all over the world. The physical dance movement is shown in Figure 1.

As shown in Figure 1, in a sports dance program, the technique and expressiveness of fully expressing dance skills are at the core of the program. For male and female athletes, it is necessary not only to perform technical movements correctly, but also to develop strength and speed, and to reflect the beauty of vitality. It also needs to convey charm through personal body language, eye contact, and tacit cooperation between dance partners. Dancers need to hone and shape the dance movements in their minds while practicing for a long time [7].

RETRACTED

With the improvement of the competitive characteristics of sports dance activities, athletes have higher and higher requirements for various basic properties of the body, which is to better complete the technical movement. As the training load increases and the difficulty of exercise continues to increase, it is easy to strain the ligaments due to exercise. Ligament injuries are undoubtedly invisible to the naked eye for athletes, and have a great impact on the usual training [8].

The common causes of sports ligament injuries are as follows:

#### 3.1.1. Training Factors

The main causes of sports injuries in sports dance training can be divided into two aspects: subjective and objective. Subjective factors mainly include athlete's lack of physical strength, lack of learning of technical necessities, and neglect of the importance of warm-up preparation [9]. Athletes need the coordination of muscles and various limbs of the whole body, which requires high physical strength, flexibility and endurance of athletes, and the risk of injury to athletes increases [10].

#### 3.1.2. Lack of Reasonable Preparation for Warm-Up Activities

The technical movements in sports dance require very high movement strength and speed. If the athlete does not have a good competition training state, the coordination of various organs of the body and the high concentration of attention will easily lead to sports injuries. Preparatory warm-up activities can effectively improve the excitability of the nervous center and the coordination of the limbs. It is very important to prepare for warm-up activities in any sports, and it is also essential in the competition and training of sports dance [11].

#### 3.1.3. Technical Errors and Mistakes

Sports dance consists of ten dance types, each of which has different technical characteristics, which makes it easy for athletes to confuse and make mistakes in training and learning. With the rapid development of the Internet, the technical routines of elite athletes have been widely disseminated, and the difficulty factor of learning their skills has also doubled when they sighed at the beautiful dance postures of athletes. This makes athletes make frequent mistakes in the process of technical training. Some wrong movements do not conform to the characteristics of human physiology. If they do not correct and develop habits in time, the possibility of injury will be greatly increased.

#### 3.1.4. Poor Physical Fitness

The physical fitness of sports dancers is not good. During the investigation of athletes, it was found that although the academy offered physical courses, athletes generally lacked basic physical fitness training and special physical fitness training. It is difficult to effectively improve the strength, explosiveness, and endurance, which is unfavorable for the development of sports dance. With the continuous development of sports dance competition toward difficulty and beauty, the competition is becoming increasingly fierce, and the athletes' poor physical fitness makes it difficult to support the technical requirements and competition intensity.

RETRACTED

### 3.2. Damage Identification Based on Deep Learning

In recent years, the rapid development of health monitoring application research has attracted the attention of many experts and scholars, and damage identification has become the core of the task of health monitoring systems [12, 13]. A major research topic in structural health monitoring is the determination of structural damage. Structural health monitoring technology was first developed in the aerospace field and was originally designed to monitor structural loads. With the development of large-scale complex and intelligent structural design, the content of structural health monitoring is gradually enriched, not only the simple load monitoring, but also the detection of structural damage and the prediction of structural life [14, 15].

Deep learning is a new research field developed on the basis of machine learning, and is the latest theoretical achievement of artificial neural networks. In recent years, it has achieved excellent results in many practical applications such as time series data prediction, speech recognition, image recognition, and computer vision [16, 17]. Deep learning is to learn the inherent laws and representation levels of sample data, and the information obtained in these learning processes is of great help to the interpretation of data such as text, images, and sounds. Its ultimate goal is to enable machines to have the ability to analyze and learn like humans, and to recognize data such as words, images, and sounds. The original intention of the deep artificial neural network is to establish a model that simulates the neurons of the human brain to simulate the working principle of the human brain. When processing time series data, images, speech, and text data, it learns data features hierarchically through multiple high-order function stages, so as to obtain effective feature representations for recognition tasks. A schematic diagram of the structure of deep learning is shown in Figure 2.

As shown in Figure 2, deep learning is currently the most popular subfield of machine learning, and its purpose is to build a trainable deep model to simulate the processing and problem analysis process of the human brain [18, 19]. The concept of deep learning comes from the detailed study of artificial neural networks, the learning of layered processing methods for visual systems, and the solution to the problem of vanishing gradients caused by too many layers of multilayer neural networks.

RETRACTED

### 3.3. Convolutional Neural Networks for Structural Health Monitoring

Firstly, the problem is discretized. In theory, neural network can be used to simulate functions of arbitrary complexity. As long as enough training data is used, a good regression model can also be obtained for functions of continuous real numbers [20, 21]. A regression model is a predictive modeling technique that studies the relationship between the dependent variable (target) and the independent variable (predictor). This technique is often used for predictive analysis, time series modeling, and finding causal relationships between variables. However, for a complex function, such as the mapping from mode shape frequency to damage value, although the neural network can theoretically be used for numerical regression, the training complexity is too high, and it is difficult to achieve in practical scenarios. The convolutional neural network is shown in Figure 3.

As shown in Figure 3, convolutional neural network is a kind of feedforward neural network with convolution calculation and deep structure, which is one of the representative algorithms of deep learning. The convolutional block is formed by stacking 4 layers of networks, which are the convolutional layer, the BatchNorm layer, the activation layer, and the Dropout layer. A convolutional layer consists of a set of feature selectors, each with its own learnable receptive field. Through the scanning of the receptive field on the input, the feature selector can only mention the information that it is interested in [22, 23]. The receptive field refers to the size of the region where the pixels of the feature map output by each layer of the convolutional neural network are mapped back to the input image. For each feature selector, its mathematical form is formula:

(1) $$\begin{array}{c} b_{i}=\sum_{l=0}^{l}\sum_{c=0}^{c}W_{l},a_{i+1}^{c}\text{.} \end{array}$$

Among them, *a*_*i*+1_^*c*^ is the *i* + *l*-th value in the *c*-th feature vector in the input, *W*_*l*_ is the corresponding weight, *b*_*i*_ is the value of the corresponding selector at the *i*th position, and *L* is the length of the receptive field [24, 25]. When scanning over the input, one length is slided at a time, and a zero is added to the beginning and end of each feature vector of the input for padding, as shown in Figure 4.

As shown in Figure 4, the BatchNorm layer achieves the purpose of accelerating model convergence by regularizing the input. Its formula is formula:

(2) $$\begin{array}{c} \mu_{B}\leftarrow \frac{1}{m}\sum_{i=1}^{m}a_{i}\text{.} \end{array}$$

The ReLU function is a general activation function that is widely used at present. The LeakyReLU function is the best choice if we encounter a situation where neurons are not activated in network. LeakyReLU is an activation function that people use to provide nonlinearity to the model and enhance the expressiveness through the activation function. Its expression is shown in the following formula:

(3) $$\begin{array}{c} f\left(a\right)=\max\;\left(0,a\right)+\lambda *\;\min\;\left(0,a\right)\text{.} \end{array}$$

Dropout, as the name suggests, means to be removed, just because we removed some neurons in the neural network, it is called the dropout layer. The Dropout layer randomly discards some features to enhance the robustness of the model and prevent the model from overfitting. Residual blocks are similar to two-layer stacked convolutional blocks, but before the last dropout layer, people add the input and the output processed by the layer-by-layer network once, and note that people in the design ensure that the output is the same as the input after the convolution block processing. Let *f*(*a*) represent the processing of the input a by the first 7 layers in the residual block, then before the dropout layer, people's operations are shown in the following formula:

(4) $$\begin{array}{c} b=f\left(a\right)+a. \end{array}$$

The eigenvalues and eigenvectors are for the matrix. Obviously, this matrix is the eigenmatrix, and each column in the eigenmatrix is a feature. Sending the feature matrix into the full connection to get the output fout of the model, where B is the weight matrix obtained by learning, and *b* is an example of the intermediate result of the bias model obtained by learning, and the output is shown in the following formula:

(5) $$\begin{array}{c} fout=f\text{eat}B+b\text{.} \end{array}$$

Argmax is a function, which is a function to obtain parameters (sets) of functions. Using argmax to get the prediction result, the function of the argmax function is to obtain the index with the largest value. The prediction result is shown in the following formula:

(6) $$\begin{array}{c} pred=\text{argmax}\left(f\text{out}\right)\text{.} \end{array}$$

Then the predicted result is divided by 1000 to get the final predicted damage value. The loss function is shown in the following formula:

(7) $$\begin{array}{c} \text{Loss}=\overset{n}{\underset{i=1}{\sum }}-\log\frac{e^{y}}{\sum_{j=1}^{c}e^{y}}\text{.} \end{array}$$

Among them, *e*^*y*^ is the output of the model for category *j*, y corresponds to the output of the model for the real category, *n* is the number of samples, and people's goal is to make Loss as small as possible. The smaller the Loss, the more accurate the model's prediction of damage values.

RETRACTED

During training, the predicted value is calculated, and the training result is minimized using the true value and gradient descent. Gradient descent is a first-order optimization algorithm, also commonly known as steepest descent. To find the local minimum of a function using gradient descent method, it is necessary to iteratively search for points with a specified step distance in the opposite direction of the gradient corresponding to the current point on the function. The parameter set that can minimize the loss is found, as shown in the following formula:

(8) $$\begin{array}{c} \theta =\text{argmin}\overset{n}{\underset{i=1}{\sum }}-\log\frac{e^{y}}{\sum_{j=1}^{c}e^{y}}\text{.} \end{array}$$

A supervised learning process detects structural damage/location as well as size. Unsupervised learning can detect damage and location, and both methods have their own advantages and disadvantages. Supervised learning needs to obtain the damage sample state of the structure through finite element simulation, but unsupervised learning does not. Supervised training requires long enough samples. Supervised learning can detect the location and size of damage, while unsupervised learning can only detect damage and location, and the accuracy is not high.

### 3.4. MLP Neural Network

Firstly, the problem is discretized. In theory, neural network can be used to simulate functions of arbitrary complexity. As long as there is enough training data, a good regression model can also be obtained for functions of continuous real numbers. The multilayer perceptron neural network model is shown in Figure 5.

As shown in Figure 5, the neuron node of MLP adopts a signal activation function, and the output value of the function changes continuously and monotonically from -1 to 1, so the mapping from any input value to the output value can be realized. In the neuron, the inputs are weighted and summed, and then a function is applied, which is the activation function. The activation function is introduced to increase the nonlinearity of the neural network model.

The weight adjustment method also uses the BP algorithm. For the Pth sample, the output of the kth hidden layer node is shown in the following formula:

(9) $$\begin{array}{c} O_{p}\left(k\right)=f\left(\overset{n+1}{\underset{n=1}{\sum }}w_{ih}\left(k,n\right)\cdot a_{p}\left(n\right)\right)\text{.} \end{array}$$

Among them, *f*(•) is the sigmoid excitation function, and the ith output *b*_*p*_(*i*) can be expressed as shown in the following formula:

(10) $$\begin{array}{c} b_{p}\left(i\right)=\overset{n+1}{\underset{n=1}{\sum }}w_{oi}\left(i,n\right)\cdot a_{p}\left(n\right)\text{.} \end{array}$$

A commonly used error function is the mean square error function, which can be expressed as shown in the following formula:

(11) $$\begin{array}{c} E=\frac{1}{N_{v}}{\overset{N_{v}}{\underset{p=1}{\sum }}\overset{M}{\underset{i=1}{\sum }}\left[t_{p}\left(i\right)-b_{p}\left(i\right)\right]}^{2}=\overset{M}{\underset{i=1}{\sum }}E\left(i\right) \end{array}$$

So the error function for each output value *b*_*p*_ is shown in the following formula:

(12) $$\begin{array}{c} E\left(i\right)=\frac{1}{N_{v}}{\overset{N_{v}}{\underset{p=1}{\sum }}\left[t_{p}\left(i\right)-b_{p}\left(i\right)\right]}^{2} \end{array}$$

The formula for calculating the gradient is as shown in the following formula:

(13) $$\begin{array}{c} g\left(m\right)=\frac{\partial E\left(i\right)}{\partial W\left(i,m\right)}=\frac{\partial E{\left(t_{i}-b_{i}\right)}^{2}}{\partial W\left(i,m\right)}\text{.} \end{array}$$

Substituting *b*_*i*_ into the above formula and simplifying yields formula:

(14) $$\begin{array}{c} g\left(m\right)=-2E\left[t_{i}-b_{i}\right]A\left(m\right)\text{.} \end{array}$$

RETRACTED

### 3.5. Health Monitoring Model Based on Multivariate Gaussian Distribution

The Gaussian distribution is also known as the normal distribution, and its corresponding probability density function can be expressed as shown in the following formula:

(15) $$\begin{array}{c} P\left(a,\mu ,\sigma^{2}\right)=\frac{1}{\sqrt{2\pi \sigma }}\exp\;-\left(\frac{{\left(a-\mu \right)}^{2}}{2\sigma^{2}}\right)\text{.} \end{array}$$

Among them, the existing data can be used to calculate *μ* and *σ*^2^ in the probability density function, and the calculation method is as shown in the following formula:

(16) $$\begin{array}{c} \mu =\frac{1}{m}\overset{m}{\underset{i=1}{\sum }}a^{\left(i\right)}\text{.} \end{array}$$

The multivariate Gaussian distribution is developed from the univariate Gaussian distribution, and is a generalization based on the univariate Gaussian distribution. It has many advantages, and this paper uses these characteristics to construct a health state assessment model. The multivariate Gaussian distribution model will be described in detail below. A random variable distribution that satisfies the following probability density distribution is called a two-dimensional normal distribution as shown in the following formula:

(17) $$\begin{array}{c} f\left(a,b\right)={\left(2\pi \sigma_{1}\sigma_{2}\sqrt{1-\rho^{2}}\right)}^{-1}\text{.} \end{array}$$

The function is a probability density function, which should satisfy the basic properties of the probability density function: one is greater than zero, and the other is that the integral over the whole space is equal to 1.

RETRACTED

The multivariate normal distribution is also called the multivariate Gaussian distribution, and the multivariate Gaussian model is an extension of the univariate Gaussian probability density function. In the multivariate Gaussian distribution model, in order to obtain the feature *a*^(*i*)^, the covariance matrix ∑_*i*=1_^*m*^*a*^(*i*)^ of the feature needs to be constructed. The specific calculation method is as shown in the following formula:

(18) $$\begin{array}{c} \mu =\frac{1}{m}\overset{m}{\underset{i=1}{\sum }}a^{\left(i\right)}\text{.} \end{array}$$

Finally, the probability value of the multivariate Gaussian distribution is calculated as shown in the following formula:

(19) $$\begin{array}{c} \rho \left(a\right)=\frac{1}{{{\left(2\pi \right)}^{n/2}\left|\Sigma \right|}^{1/2}}\text{.} \end{array}$$

Among them, *μ* is a vector, each cell of which is the mean of a row of data in the original matrix.

## 4. Ligament Repair Experiment Based on Health Monitoring

### 4.1. Experiments on the Accuracy of Neural Networks and Gaussian Distributions

#### 4.1.1. Experiments on Convolutional Neural Networks and MLP Neural Networks

In the feature extraction stage, this paper applies a deep neural network consisting of two convolutional layers and two downsampling layers to learn the features of the original signal. When training the parameters of the network, the optimal parameter combination of the network is obtained through continuous iteration and trial. In the health status assessment stage, the features learned by the convolutional neural network are applied to the multivariate Gaussian distribution. First, the multivariate Gaussian model is used to obtain the probability distribution of the features. Then, it is divided into different probability intervals, and some feature points in the small probability interval are considered as a feature representation of a healthy state. The feature points in different probability intervals are divided into health status grades according to the size mark of the probability mean value of the interval feature points [26, 27].

The MLP neural network is also a multilayer perceptron, which is used for feature fusion. Each neuron has its own weight, and there are many parameters, which are updated during backpropagation. Using the Relu activation function in the experiments, the number of iterations of the MLP neural network model is 80. The change of MLP training accuracy and the change of time are shown in Figure 6.

RETRACTED

As shown in Figure 6, it can be inferred from this that the initial parameter setting of the model is reasonable, and there is no over-adaptation phenomenon of training. After the model is trained, the training of the model can be stopped. The runtime of the accurate model can be obtained from the runtime curve. The performance of the model is evaluated with the test set, and the changes in MLP test accuracy and aging are shown in Figure 7.

As shown in Figure 7, the method of MLP neural network is relatively simple, and the training speed is relatively fast. The MLP neural network is connected by neurons, and the parallelism of MLP becomes high. It can also be seen that the MLP test accuracy becomes higher and higher as the number of iterations increases.

#### 4.1.2. Gaussian Distribution

In this paper, the original physiological signal features learned by the convolutional neural network are provided to the multivariate Gaussian health state assessment model [28, 29].

In order to make the reconstruction error converge when adjusting the network weights, before sending the original signal to the convolutional neural network, it is also necessary to normalize the original signal of different dimensions, as shown in the following formula:

(20) $$\begin{array}{c} A_{\text{norm}}=\frac{a-mu}{std\left(a\right)}\text{.} \end{array}$$

*mu* and *std*(*a*) represent the mean and standard deviation of the original signal, respectively. The normalized standard signal is then fed to the convolutional neural network to learn the features of the signal. By analyzing the relationship between the reconstruction error and the number of iterations between the original signal and the reconstructed signal, a set of relatively good characteristics of the original signal can be obtained.

In data modeling, the multivariate Gaussian distribution model is often used, and when it is extended to multidimensional data, the multivariate Gaussian distribution is used to describe it. When the features are learned from the original signal and provided to the multivariate Gaussian model for health assessment, it is also necessary to consider whether the learned features conform to the Gaussian distribution. The Gaussian distribution of features under different samples is shown in Figure 8.

As shown in Figure 8, the Gaussian distribution of the six athletes' physiological signal characteristics has been calculated to verify whether it conforms to the Gaussian distribution. It is intuitive to see that the six athletes' physiological signal characteristics obtained in this experiment conform to the Gaussian distribution.

To study the recognition situation of using convolutional neural network algorithm, under the assumption of uniform distribution of damage probability of each unit, from the analysis of the accuracy of damage recognition of each unit, the analysis of the accuracy of damage recognition of all units, and the analysis of the accuracy of structure record. The unit accuracy analysis mainly evaluates the distribution of the structural damage identification accuracy of each unit under different error conditions, as shown in Figure 9.

RETRACTED

As shown in Figure 9, it can be clearly seen that the prediction results of each point obtained by using the single-point model are similar, which successfully overcomes the shortcomings of low accuracy of some detected points. Good results have been achieved at each measurement point. Unit deep learning is used for structural health monitoring, and the required algorithm model can be selected according to different precision scenarios.

### 4.2. Investigation of Ligament Injury in Sports Dancers

The findings of this study show that among the 120 athletes participating, there are four categories of competitors: men's Latin, men's standard, women's Latin, and women's standard. Latin male and female players account for a larger proportion, as shown in Table 1.

As shown in Table 1, the number of women's Latinos is 40, the largest number and the largest proportion, and the number of men's Latinos ranks second, with 35 people, and all athletes are under 30 years old.

Sports injuries can be divided into mild, moderate, and severe injuries according to their degree. In this article, it is divided according to the length of time that cannot participate in sports after the injury, as shown in Table 2.

As shown in Table 2, sports injuries are divided into mild, moderate, and severe injuries. Among them, the number of minor injuries is 20, accounting for 16.7%. Severe injury was 45 people, accounting for 37.5%, and moderate injury was 55 people, accounting for 45.8%. It can be seen that the number of people with moderate ligament injury is the largest, and the ranking is also the first, so ligament injury should not be ignored.

This paper also investigates the main symptoms of dance sports injuries, as shown in Table 3.

As shown in Table 3, among dance sports injuries, ankle ligament injuries, medial and lateral knee ligament strains, lumbar muscle strains, toe joint strains, shoulder deltoid strains, and other injuries were investigated. Ankle ligament injuries were found in the largest number of people. According to the nature of injury, 120 sports dancers were counted, including 50 males and 70 females.

In order to verify the authenticity of the experiment, this paper investigates and analyzes the prevalence of sports injuries among sports dancers of different genders, as shown in Table 4.

RETRACTED

As shown in Table 4, a higher percentage of ligament injuries occurred in female athletes than in male athletes. Women's movement techniques are more complex and changeable, so the injury rate of women is higher than that of men.

This article also investigates the measures athletes take after ligament injuries, as shown in Table 5.

As shown in Table 5, among the contestants in this survey, less than half of the contestants had joint injuries and required surgery. Analysis of various treatment methods shows that arthroscopy has higher accuracy in reflecting intra-articular conditions, and has relatively few postoperative complications, basically does not affect the surrounding muscle structure, and can function exercise earlier after surgery. Therefore, arthroscopy has become the first choice for the diagnosis and treatment of joint injuries.

### 4.3. Recovery and Treatment of Ligament Injury after Competition Training

#### 4.3.1. Massage to Relax

By massaging the joints, the elasticity of the ligaments can be enhanced, and the range of motion of the joints can be increased, especially for the injured joints, ligaments, and muscle bonds, which can greatly speed up the recovery effect. When massage is relaxed, it can choose to focus on the parts that are easily damaged in sports dance, such as: soleus, gastrocnemius, and quadriceps of the lower limbs in Latin dance. It can also massage and relax the fatigued parts according to the proprioception. When sports dancers feel very tired, they need to massage the muscles and joints of the whole body to relax.

For mild ligament injury, quickly apply ice cubes or cold water to rinse after the injury, and then apply pressure bandage, elevate the injured foot as much as possible when resting or sleeping. After 24 hours, massage the injured ankle, apply heat with a towel, and apply safflower oil and other medicines to increase blood circulation and speed up swelling.

#### 4.3.2. Reasonably Arrange the Training Load

In the arrangement of training volume, attention should be paid to the organic combination of large, medium, and small, so as to achieve step-by-step progress, and to formulate personalized training and competition plans based on the rationale and physiological characteristics of individual players. However, the actual situation is that the training volume of athletes is often arranged closely within a period of time, such as during class, which leads to excessive load on local muscles. Or if two consecutive training sessions are repeated with the same form of force, the burden of local muscles will inevitably increase under the condition of repeated force, resulting in the occurrence of sports injuries. Therefore, the scientific nature of training is very important. Blindly greed for more and eager for success are the direct causes of sports injuries.

RETRACTED

#### 4.3.3. Reasonable and Adequate Preparation Activities

The preparatory activities for sports dance should consist of freehand exercises, stretching exercises, and basic step exercises. The intensity of the warm-up preparation activities should be controlled at low to moderate intensity, and the athlete should feel the body warm and sweat slightly, and not make the body feel tired. According to the characteristics of sports dance, the daily training warm-up preparation time should be controlled at about 10 minutes, and the competition should be prepared according to the actual situation, athletes participating in the dance, weather factors, and other targeted preparations.

## 5. Conclusions

As sports dance programs are gradually becoming known to the world, the demand for professionals in the field of sports dance is also increasing. According to the needs of social development, sports art colleges and universities have successively opened sports dance majors, and the number of sports dance experts in the team has continued to increase. However, in dance sports, many athletes will suffer from ligament strain due to the need for limb flexibility and technical tests. Therefore, this paper studies the repair of ligament strain based on health monitoring. In the method part, based on health monitoring, this paper proposes a deep learning algorithm. Deep learning has the function of damage identification. On the basis of deep learning, convolutional neural network, MLP neural network, and Gaussian distribution are proposed. In order to verify the accuracy of the MLP neural network, this paper explores it in the experimental part, and finally found that the accuracy of the MLP neural network is high. Then a survey of 120 sports dancers was conducted, and it was found that most of them would cause injuries during sports. No matter what kind of dance, the probability of ligament strain was the greatest. Finallthis paper puts forward some suggestions for the factors of ligament strain. After all, the author's ability is limited, and there are still many areas for improvement in the experimental part. The author will definitely work harder in the future.

## Figures and Tables

**Figure 1:** Sports dance movement.

**Figure 2:** Deep learning architecture.

**Figure 3:** Convolutional neural network.

**Figure 4:** Example of a convolutional layer.

**Figure 5:** Multilayer perceptron neural network model.

RETRACTED

**Figure 6:** Comparison of MLP training accuracy changes and aging changes. (a) MLP training accuracy curve, and (b) MLP training running time curve.

**Figure 7:** Comparison of MLP test accuracy changes and aging changes. (a) MLP test accuracy curve, and (b) MLP test running time curve.

**Figure 8:** Six athlete physiological signal characteristics.

**Figure 9:** Distribution of structural damage identification accuracy under different samples.

**Table 1:** The situation of male and female dancers of different dance styles.

Dance	Number of people	Age	Height (cm)	Weight (kg)
Latin male	35	21–25	177–180	63–65
Standard male	20	18–25	178–182	62–65
Latin woman	40	15–27	165–175	42–50
Standard female	25	18–22	166–172	45–52

**Table 2:** Injury degree questionnaire for sports dancers.

Hurt	Number of people	Percentage (%)
Minor injury	20	16.7
Moderate damage	55	45.8
Severe injury	45	37.5

**Table 3:** Main symptoms of sports dance injury.

Specific injury	Number of people	Percentage (%)
Ankle ligament injury	36	30
Knee medial and lateral ligament strain	32	26
Lumbar muscle strain	20	17
Toe joint strain	16	13.3
Shoulder deltoid strain	9	7.5
Other	7	6.2

**Table 4:** Prevalence of sports injuries in sports dancers of different genders.

Gender	Number of people surveyed	Injured	Percentage (%)
Male	50	38	76
Female	70	61	87
Total	120	99	163

**Table 5:** Actions taken by athletes after ligament injury.

Measure	Number of people	Percentage (%)
No joint surgery	68	57
Diagnostic joint endoscopy	21	17.5
Surgical joint endoscopy	12	10
Arthrotomy	10	8.3
Other operations	9	7.2

## Data Availability

The data that support the findings of this study are available from the corresponding author upon reasonable request.
